# Significance of Edaravone Combined with Emotion Management Model in Promoting the Recovery Process and Improving Negative Psychology in Patients with Type 2 Diabetes Mellitus Combined with Stroke

This article has been retracted.

**DOI:** 10.1155/2022/8099997

**Published:** 2022-10-10

**Authors:** Xiaoyun Lv, Xiaolan Lu

**Affiliations:** ^1^Department of Nephrology, Taicang Hospital of Traditional Chinese Medicine, Suzhou, Jiangsu 215400, China; ^2^Department of Encephalopathy, Taicang Hospital of Traditional Chinese Medicine, Suzhou, Jiangsu 215400, China

## Abstract

**Methods:**

Eighty-one patients with T2DM combined with CS who attended our hospital and received rehabilitation treatment from March 2020 to May 2021 were enrolled to a prospective nonrandomized controlled analysis. Among them, 46 patients received EDA combined with emotional management model and were regarded as the observation group (OG), and 35 received EDA combined with conventional care and were seen as the control group (CG). The clinical efficacy and glycemic function of the two groups were compared, and the scores of the Activities of Daily Living (ADL), Pittsburgh Sleep Quality Index (PSQI), and Self-Assessment Scale for Anxiety and Depression (SAS and SDS) were investigated before and after treatment. At the time of discharge, patient satisfaction with care was counted. Within six months after prognosis, T2DM self-management behavior and CS self-management behavior score surveys were conducted.

**Results:**

There was no difference in clinical efficacy between both groups (*P* > 0.05); The posttreatment glucose, PSQI, SAS, and SDS scores were lower in the OG than in the CG, while ADL and emotional management scores were higher than in the CG (*P* < 0.05). In addition, both nursing satisfaction and prognosis disease self-management behavior scores were also higher in the OG than in the CG (*P* < 0.05).

**Conclusion:**

The EDA combined with emotion management model can effectively promote the recovery process of patients with type II T2DM combined with CS, while improving their negative psychology and enhancing their self-management ability, which has high potential for clinical application.

## 1. Introduction

Diabetes is a group of metabolic diseases characterized by hyperglycemia, the incidence of which continues to rise with the aging of the population and changes in lifestyle [1]. Diabetes mainly consists of type 1 and type 2 (T2DM), with T2DM accounting for 90 to 95% of all diagnosed T2DM cases [2]. Currently, T2DM cannot be cured and requires long-term drug control, but prolonged disease is likely to cause multisystem damage, leading to chronic progressive lesions and hypofunction of multiple organs, threatening the life and health of patients [3]. Cerebral stroke (CS) is a common complication of T2DM, caused by obstruction of blood circulation in the brain; its morbidity and mortality rates are much higher than those of other brain injury diseases, and the disability rate is increasing [4, 5]. Therefore, facing patients with T2DM combined with CS requires not only effective pharmacological control but also improving patient self-management, safeguarding patients' recovery process, and promoting a positive mindset are crucial for disease treatment [6].

Edaravone (EDA) is a brain protective agent commonly used in the clinic practice to scavenge free radicals and inhibit lipid peroxidation and has achieved excellent results in improving neurological symptoms, activities of daily living, functional impairment, ischemic cerebrovascular disease, and muscular dystrophy spinal cord sclerosis due to acute cerebral infarction [7, 8]. For CS, EDA has also been shown to have excellent results, but studies have not been conducted in detail for patients with combined T2DM among them [9, 10]. It remains unclear whether the presence of T2DM negatively affects the treatment of EDA. What is more, in modern clinical treatment of patients with T2DM combined with CS, the treatment of patients is no longer limited to the improvement of the pathological content, but also needs to improve their psychology, self-management, and quality of life in many aspects [11]. More targeted and personalized care measures play a decisive role in this process [12]. Emotion management model of care program is a personalized care focused on the changes of patients' psychology, which has achieved excellent results in the treatment of various cancer diseases [13, 14], but its effectiveness in patients with T2DM combined with CS still lacks research corroboration.

In the present study, we collected 81 patients with T2DM combined with CS who attended our hospital and received rehabilitation treatment from March 2020 to May 2021 to a prospective nonrandomized controlled analysis, and divided them into 2 groups. Then, we investigated the effect of EDA combined with emotion management model on patients with T2DM combined with CS.

## 2. Materials and Methods

### 2.1. Study Area

The study was carried form March 2020 to January 2022.

### 2.2. Patients' Clinical Data

Eighty-one patients with T2DM combined with CS who attended our hospital and received rehabilitation treatment from March 2020 to May 2021 were enrolled to a prospective nonrandomized controlled analysis, including 47 males and 34 females, with an average age of 58.2 ± 14.5 years. Among them, 46 patients received EDA combined with emotional management model and were regarded as the observation group (OG), and 35 received EDA combined with conventional care and were seen as the control group (CG).

### 2.3. Inclusion and Exclusion Criteria

Inclusion criteria: laboratory tests at our hospital consistent with a confirmed diagnosis of T2DM with CS; complete clinical profiles of patients, with telephone follow up available; patients were in stable condition, without serious complications including liver or kidney dysfunction, myocardial infarction, heart failure, respiratory failure, or pulmonary infection; no cerebral hemorrhage; the patient and family volunteered to take part in this study, and the compliance was good. The study was conducted with the approval of the Medical Ethics Committee, and all patients were informed and signed an informed consent form. Exclusion criteria: persons with drug contraindications; patients with severe liver and kidney insufficiency, combined with other malignancies; patients with severe cardiovascular and cerebrovascular diseases; patients with severe inflammation; pregnant or lactating women.

### 2.4. Methods

The CG received EDA combined with conventional care treatment: patients were admitted to the hospital and received conventional treatment such as controlling blood glucose, blood pressure, improving blood circulation and promoting neurological recovery, etc. On top of this, they received EDA treatment, 30 mg of EDA diluted in an appropriate amount of saline and administered intravenously within 30 min, twice daily for 14 d. Besides, the medical staff assisted the patients to do a series of examinations after admission, explained the need for precautions, observed their conditions, monitored the fasting, postprandial blood glucose two hours after lunch and dinner, understood their conditions and made timely records, and provided dietary intervention and rehabilitation training. The OG was treated with EDA combined with an emotion management model: the EDA treatment was the same as the CG, and the emotional management model was implemented on this basis to explain disease-related knowledge and classic cases to patients to enhance their treatment confidence and promote compliance. Health education was implemented to inform patients and their families of the purpose of care and the importance of medication, to properly guide patients to self-control, to establish confidence in treatment and health goals, and to help them to perform appropriate exercises to improve their daily living skills. Patients were given positive encouragement to help them establish a correct and positive attitude toward treatment, and timely interventions were made for their psychological adverse emotions, including listening to soothing music to relax their bodies and minds and improve their psychology. Nursing staff need to strictly control patients' daily meal fat intake and sugar, to ensure that their nutrition is balanced, to give more affirmation and encouragement to them, targeted to provide meticulous care to accelerate their recovery.

### 2.5. Outcome Measures

*(1) Clinical Outcomes*. The cases were divided into basic cure (symptoms were basically controlled and more stable), improvement (symptoms were greatly improved), progress (symptoms were improved but the condition was still unstable), and ineffective (treatment had no effect), and the total effective rate = (basic cure + improvement)/total number of cases × 100%.

*(2) Blood Glucose Function*. Fasting venous blood was drawn before and after treatment and sent to our laboratory to check fasting blood glucose (FBG) and 2-hour postprandial blood glucose (2hPG).

*(3) Life Situation*. Pre and posttreatment assessments were made using the Activities of Daily Living (ADL) scale (higher scores indicate greater ability to perform activities of daily living) and the Pittsburgh Sleep Quality Index (PSQI) (lower scores indicate better sleep quality). For ADL score, a total score of 0 indicated total dependence and a score of 100 indicated full independence. Besides, severe dependence (0–40), moderate dependence (41–60), and mild dependence (61–99). The total score of PSQI was 21. For this study, we used PSQI > 5 as an indicator of sleep disorder, and PSQI> score 10 as severe sleep disorder.

*(4) Psychology*. Anxiety and depression self-assessment scales (SAS and SDS) were used to assess psychology of patients before and after treatment, with lower scores indicating greater psychological health. The index score of SAS was no anxiety ( <50); low anxiety (50~59); moderate anxiety (60~69), and severe anxiety ( > =70), the index score of SDS was no depression ( <50); low depression (50~59); moderate depression (60~69), and severe depression ( > =70).

*(5) Emotion Management*. Our self-made emotion management ability scale was used to assess three dimensions: mental activity management, partnership, and emotion processing, with higher scores indicating better emotion management ability.

*(6) Nursing Satisfaction*. When patients were discharged from the hospital, a nursing satisfaction survey was conducted, which was divided into four levels: very satisfied, satisfied, to be improved, and unsatisfied.

*(7) Six Months of Prognosis*. Patients were surveyed for disease self-management behavior scores (including T2DM and CS), with higher score results indicating greater self-control.

### 2.6. Statistical Methods

The data were statistically analyzed by SPSS 24.0 statistical software, and the experimental results were recorded in the form of (mean ± standard deviation) by calculating the mean. Comparisons between groups were made using independent samples *t*-tests, and paired *t*-tests were used before and after treatment. Statistically remarkable differences were considered when *P* < 0.05.

## 3. Results

### 3.1. Comparison of Treatment Results between Two Groups of Patients

In the OG, the basic cure rate was 34.78%; the improvement rate was 39.13%; the progress rate was 21.74%; the invalidity rate was 4.35%, and the total effective rate was 73.91%. In the CG, the basic cure rate was 34.29%; the improvement rate was 34.29%; the progress rate was 22.86%, and the invalidity rate was 8.57%, with an overall effective rate of 68.57%. There was no statistically obvious difference in the total effective rate of treatment between groups (*P* > 0.05, Table 1).

### 3.2. Comparison of Blood Glucose Levels between Groups before and after Treatment

Before treatment, there was no difference in BG compared with 2hPG in both groups (*P* > 0.05), while BG was (6.45 ± 1.85) mmol/L in the OG after treatment, which was even lower than BG (7.25 ± 1.91) mmol/L in the CG after treatment (*P* < 0.05, Figure 1(a)). The 2hPG in the OG was (8.91 ± 1.45) mmol/L, which was also lower than that in the CG (*P* < 0.05, Figure 1(b)).

### 3.3. ADL and PSQI Scores before and after Treatment

No significant differences were seen in ADL and PSQI scores between both groups before treatment (*P* > 0.05). ADL score was increased after treatment in two groups, and ADL score in OG was higher than that in CG (*P* < 0.05, Figure 2(a)). PSQI score was decreased after treatment in two groups, and PSQI score in OG (7.15 ± 1.25) was lower than that in the CG (8.86 ± 1.44) (*P* < 0.05, Figure 2(b)).

### 3.4. SAS and SDS Scores before and after Treatment

Before treatment, the differences in SAS and SDS scores between both groups were not statistically marked (*P* > 0.05). After treatment, the SAS score of the OG was (32.63 ± 1.58), which was lower than that of the CG (*P* < 0.05, Figure 3(a)). After treatment, the observed SDS score in the OG was (32.72 ± 1.53), which was also lower than that of the CG (*P* < 0.05, Figure 3(b)). SAS and SDS scores were dramatically lower in both groups after treatment than before treatment (*P* < 0.05).

### 3.5. Emotion Management Ability Score before and after Treatment

After treatment, the emotional management ability scores of both groups were dramatically higher (*P* < 0.05) than those before treatment. The mental activity score of OG (57.76 ± 3.59) was higher than that of the CG (46.17 ± 2.51) (*P* < 0.05, Figure 4(a)). The partnership score in OG (56.22 ± 3.06) was higher than that in CG (45.86 ± 3.45) (*P* < 0.05, Figure 4(b)). It was seen that the emotional processing score was in OG (57.02 ± 4.56), which was also higher than that in CG (*P* < 0.05, Figure 4(c)).

### 3.6. Prognosis Self-Management Score

Six months after discharge, the T2DM self-management behavior score of patients in the OG was (9.26 ± 1.04), which was higher than that of the CG (*P* < 0.05, Figure 5(a)). And the score of CS self-management behavior in the OG was (9.26 ± 0.98), which was similarly higher than that in the CG (6.77 ± 0.77) (*P* < 0.05, Figure 5(b)).

### 3.7. Comparison of Nursing Satisfaction

With regard to nursing satisfaction, the number of very satisfied in the OG was 58.70%, which was dramatically more than that of CG (*P* < 0.05). In addition, there were no unsatisfied patients in the OG (0.00%), while the number of unsatisfied patients in the CG was 8.57%, which was higher than that in OG (*P* < 0.05, Table 2).

## 4. Discussion

T2DM is currently the most prevalent chronic disease worldwide, which basically does not have substantial harm in itself, but is highly susceptible to causing malignant lesions in various parts of the organ tissues of the body, thus endangering the normal life and even the life safety of patients [15]. And CS is also one of the most prevalent risk factors as one of the high prevalence diseases in cardiovascular diseases, T2DM that is [16]. According to statistics, more than 60% of CS patients have an underlying disease that includes T2DM [17]. Therefore, an in-depth exploration of the treatment options for such patients has important clinical implications. In addition, because there is no cure for T2DM combined with CS, long-term medication tends to aggravate patients' negative emotions and has a great impact on their condition [18]. In contrast, the emotion management model can help patients with emotional control by enhancing their motivation for treatment, guiding them properly, and taking diverse approaches, which may be effective in alleviating their negative psychology [19]. This is important for enhancing both the effectiveness of the treatment and the prognosis of patients.

As reported previously, EDA, a novel neuroprotective agent, is a promising therapeutic strategy for the treatment of acute ischaemic stroke [20, 21]. In the present trial, we found that the total treatment efficiency of patients could reach about 70% after treatment with EDA, which was an ideal effect for patients with T2DM combined with CS [19]. Secondly, patients in both groups showed marked improvements in glycemic function, mobility, and sleep quality after treatment, which also suggested that our EDA not only had excellent effects on the disease of CS, but also could stably control patients' blood glucose and reduce the threat caused by T2DM. EDA has a reducing effect on the accumulation of hydrogen peroxide, hydroxyl, and superoxide anion groups in the body and can have an inhibitory effect on unsaturated fatty acid peroxidation and fatty acids (free radical-mediated), thus stabilizing the cell membrane state and promoting the restoration of neural function [22–24]. Therefore, in the treatment of CS, EDA can also improve patients' blood glucose function more effectively by inhibiting the oxidative stress response within the body [25]. It was seen that the treatment glycemic function, ADL, and PSQI scores were more excellent in the OG, then suggesting that we could more effectively enhance patients' treatment outcome by implementing an emotional management model during EDA treatment. We believe that the reasons for the differences between patients may be as follows: (1) Through the form of psychological counselling, the communication between patients and medical staff is increased, and patients' trust in medical staff is enhanced, which is more conducive to carrying out targeted psychological counselling and improving their anxiety, depression, and other adverse emotions [26]. This was verified by comparing the SAS and SDS scores between groups, which were lower in the OG. (2) Diversified medical activities such as psychological guidance, communication, and knowledge competitions can enrich the otherwise boring and dull inpatient life, make patients look forward to life, increase their confidence in the treatment of the disease, and be more positive in their communication with other patients and medical staff, which is of great benefit to treatment [27]. This could be verified by the fact that the ability to manage emotions improved in both groups after treatment and was higher in the OG. (3) Emotion management based on health knowledge and rehabilitation training guidance can be more effective in allowing patients to acquire and accept understanding of the disease and related knowledge, which not only improves patients' treatment compliance and treatment confidence but also allows them to have a higher degree of knowledge about their disease after discharge, improves self-management of the disease, and reduces the prognostic threat of the disease [28]. Because of this, patients in the OG had better self-management score results than the CG, including mental activity management scores, partnership scores, and emotional processing score. Ultimately, increased patient satisfaction for nursing was the expected outcome, which once again fully illustrates the value of the important application of the emotion management model in EDA treatment.

Nevertheless, we need to follow the patients for a longer period so as to find the long-term prognostic impact of the EDA and emotion management model on them. Furthermore, there may still be room for improvement in the implementation of this care strategy, as there is still a lack of uniform guidelines for the application of the emotion management model. Besides, we also need to conduct randomized controlled trials as soon as possible to compare the effectiveness of the application of the emotion management model with other care strategies to further confirm its application.

## 5. Conclusion

The EDA combined with emotion management model can effectively promote the recovery process of patients with type II T2DM combined with CS, while improving their negative psychology and enhancing their self-management ability, which has high potential for clinical application.

## Figures and Tables

**Figure 1:** Comparison of blood glucose levels between groups before and after treatment. (a) Comparison of BG between groups before and after treatment. (b) Comparison of 2hPG between groups before and after treatment. ∗ indicates that there is a statistically significant difference compared with before treatment (*P* < 0.05); # indicates that there is a statistically significant difference between the observation group and the observation group (*P* < 0.05).

**Figure 2:** ADL and PSQI scores before and after treatment. (a) Comparison of ADL scores between groups before and after treatment. (b) Comparison of PSQI scores between groups before and after treatment. ∗ indicates that there is a statistically significant difference compared with before treatment (*P* < 0.05); # indicates that there is a statistically significant difference between the observation group and the observation group (*P* < 0.05).

**Figure 3:** SAS and SDS scores before and after treatment. (a) Comparison of SAS scores between groups before and after treatment. (b) Comparison of SDS scores between groups before and after treatment. ∗ indicates that there is a statistically significant difference compared with before treatment (*P* < 0.05); # indicates that there is a statistically significant difference between the observation group and the observation group (*P* < 0.05).

**Figure 4:** Emotion management ability score before and after treatment. (a) Comparison of mental activity management scores between groups. (b) Comparison of partnership scores between groups. (c) Comparison of emotional processing scores between groups. ∗ indicates that there is a statistically significant difference compared with before treatment (*P* < 0.05); # indicates that there is a statistically significant difference between the observation group and the observation group (*P* < 0.05).

**Figure 5:** Prognosis self-management score. (a) Comparison of T2DM self-management behavior scores. (b) Comparison of CS self-management behavior scores. ∗ indicates that the difference between the two groups is statistically significant (*P* < 0.05).

**Table 1:** Clinical efficacy table.

Group	*n*	Basic cure	Improvement	Progress	Ineffective	Total effective rate
Observation group	46	16 (34.78%)	18 (39.13%)	10 (21.74%)	2 (4.35%)	34 (73.91%)
Control group	35	12 (34.29%)	12 (34.29%)	8 (22.86%)	3 (8.57%)	24 (68.57%)
*χ* ^2^						0.279
*P*						0.597

**Table 2:** Nursing satisfaction survey results.

Group	*n*	Very satisfied	Satisfied	To be improved	Unsatisfied.
Observation group	46	27 (58.70%)	16 (34.78%)	3 (6.52%)	0 (0.00%)
Control group	35	11 (31.43%)	15 (42.86%)	6 (17.14%)	3 (8.57%)
*χ* ^2^		5.934	0.549	2.270	4.095
*P*		0.015	0.459	0.132	0.043

## Data Availability

The data appearing in this article can be obtained from the corresponding author.
